# Zipper Is Necessary for Branching Morphogenesis of the Terminal Cells in the *Drosophila melanogaster*’s Tracheal System

This article has been retracted.

**DOI:** 10.3390/biology10080729

**Published:** 2021-07-30

**Authors:** Jong-Hyeon Shin, Chan-Woo Jeong

**Affiliations:** 1 Department of Molecular Biology, Princeton University, Princeton, NJ 08544, USA; 2 Department of Medicine, Seoul National University, Gwanak-gu, Seoul 08826, Korea; happysmile@jfclinic.com

**Keywords:** branching morphogenesis, seamless tube formation, zipper, tracheal system, terminal cells

## Abstract

**Simple Summary:**

The *Drosophila melanogaster*, also commonly known as the fruit fly, has a relatively simple structure, allowing scientists to study its anatomy. This research was carried out to investigate how a protein called Zipper may be important for the development of the model organism during the early developmental stages. The study concentrated on the respiratory system, also known as the tracheal system, more specifically the leading cells in the tracheal system also known as terminal cells. Zipper was shown to be in the cytoplasm of terminal cells, indicating that it may function in the *D. melanogaster*’s tracheal system. Then, comparisons between normal fruit flies and those engineered so that the RNA for *zipper* does not function were made. Visual and quantitative comparisons demonstrated less branching of the terminal cells for the mutants, while no differences were found for lumenogenesis—tube formation within the branched structures. Therefore, this study demonstrates the role of Zipper in branching of the terminal cells in the *D. melanogaster*’s tracheal system. This study adds onto the existing scientific literature by demonstrating the role of a specific protein in an important biological process occurring in most living organisms.

**Abstract:**

Branching morphogenesis and seamless tube formation in *Drosophila melanogaster* are essential for the development of vascular and tracheal systems, and instructive in studying complex branched structures such as human organs. Zipper is a myosin II’s actin-binding heavy chain; hence, it is important for contracting actin, cell proliferation, and cell sheet adhesion for branching of the tracheal system in post-larval development of the *D. melanogaster*. Nevertheless, the specific role of Zipper in the larva is still in question. This paper intended to investigate the specific role of Zipper in branching morphogenesis and lumenogenesis in early developmental stages. It did so by checking the localization of the protein in the cytoplasm of the terminal cells and also by analyzing the morphology of *zipper* RNAi loss-of-function mutants in regard to branching and lumen formation in the terminal cells. A rescue experiment of RNAi mutants was also performed to check the sufficiency of Zipper in branching morphogenesis. Confocal imaging showed the localization of Zipper in the cytoplasm of the terminal cells, and respective quantitative analyses demonstrated that *zipper* RNAi terminal cells develop significantly fewer branches. Such a result hinted that Zipper is required for the regulation of branching in the terminal cells of *D. melanogaster*. Nevertheless, Zipper is not significantly involved in the formation of seamless tubes. One hypothesis is that Zipper’s contractility at the lateral epidermis’ leading edge allows cell sheet movement and respective elongation; as a result of such an elongation, further branching may occur in the elongated region of the cell, hence defining branching morphogenesis in the terminal cells of the tracheal system.

## 1. Introduction

Branching morphogenesis and lumenogenesis are essential processes that regulate the formation of the human nervous, respiratory, and vascular systems [1,2]. Branching morphogenesis is the main process that allows the remodeling of epithelial and/or endothelial sheathes into multicellular tubular networks, ultimately allowing the transport and distribution of essential gases and metabolites, including oxygen [3]. That said, it is not surprising that mutations in genes that regulate branching morphogenesis cause defects in the kidney [4], lung [5], brain [6], and other organs in the human body. In order to learn more about the mechanism behind branching morphogenesis, as well as lumenogenesis, the research was concentrated on the larval terminal cells of *Drosophila melanogaster*’s tracheal system, which is an ideal model system as its morphogenesis and tubulogenesis have parallels to vertebrate vasculature and human genetics [7,8,9].

Branching in the terminal cells of *D. melanogaster* heavily relies on cell migration, a mechanism regulated by Branchless (Bnl), which is a fibroblast growth factor (FGF) ligand [3]. The direction of migration and, therefore, elongation of the tracheal cells is determined by the sensing of Bnl by a FGF receptor known as Breathless (Btl) [10]. This ligand–receptor interaction leads to the formation of numerous filopodia, which are within the cell that protrude and bud toward the targeted area. Hence, the Branchless–Breathless ligand–receptor signaling response allows the migration of tip cells, which is then extended further by the corresponding actin cytoskeletons [11].

Following the branching morphogenesis in the tracheal system, it is essential to form lumen via epithelial and endothelial tubes within these branched structures primarily for the transport of gases such as oxygen [12,13,14]. In the *D. melanogaster*’s tracheal system, there are three distinct layers of branching and lumen formation. The primary branches are paired with multicellular tube formation by cell migration, while secondary branches are paired with unicellular tube formation within individual tracheal cells. In addition, as discussed in this paper, terminal branches form subcellular, “seamless” tubes [15].

Most tracheal cells form “seamed tubes,” which are tubes formed as a sheet of cells roll into a tube to create distinct junctions. Uniquely, fusion cells and terminal cells make subcellular “seamless” tubes, which are tubes formed within each cell without the formation of cellular junctions. This means that the lumen network within the tracheal system is formed when single seamless tubes cooperatively generate a comprehensive lumen network throughout the entire cell [15,16].

As interesting as this seamless tube formation in the tracheal system of the *D. melanogaster* sounds, the exact mechanism is still in question. One contemporary idea is that seamless tubes are formed from a cell hollowing mechanism, where cytoplasmic vesicles fuse and form an internal tube of apical membranes that extends internally [14]. This mechanism incorporates the idea of apical–basal polarity, actin and microtubule cytoskeletal organization, cytoplasmic vesicle trafficking, and early endocytosis [17,18,19,20,21]. Some evidence supporting this mechanism is that the luminal membrane was found to be rich in apical membrane markers, actin filaments, and polarized microtubule cytoskeletons, all of which are important for the minus-end-directed transport of vesicles to form seamless tubes [13]. Furthermore, the under-production of proteins required for early endosome formation, including Rab5, Vps45, and Rabenosyn-5, formed defective cysts in the lumen, suggesting that early endocytosis is also required for proper lumen formation [4].

Nevertheless, the holistic mechanism as to how lumen formation, and branching, occurs in the tracheal system of the *D. melanogaster* still remains unclear, hence begging the question as to which specific genes are responsible for these two imperative processes in the development of the terminal cells in the tracheal system of the model organism.

It is known that the Branchless–Breathless ligand–receptor interaction leads to the formation and activation of filopodia, which are the leading extensions of actin filaments allowing the migration of tip cells [10]. The actin filaments require Zipper, an actin-binding heavy chain of nonmuscle myosin II. This is because myosin II generally has actin cross-linking and contractile properties, hence playing a contributing role in cell adhesion and migration [22,23]. What this suggests is that the Branchless–Breathless signaling pathway may ultimately lead to the actin–Zipper interaction, which is necessary for the elongation of the tracheal systems. As a result of such an elongation, branching follows in the extended region of the tracheal cell.

In order to test and justify the specific role of Zipper in branching morphogenesis, and perhaps seamless tube formation as well, it was important to first incorporate methods of cell biology to check the localization of Zipper. Sequentially, it was also important to genetically compare the morphology of *zipper* RNAi loss-of-function mutants with controls in regard to branching morphogenesis and lumenogenesis both qualitatively and quantitively. With all the results accumulated, it is logical to state that the gene *zipper* is required for regulating branching morphogenesis of the terminal cells in the *D. melanogaster*’s tracheal system, while such a gene does not play a significant role in the regulation of seamless tube formation.

## 2. Materials and Methods

### 2.1. D. melanogaster Strain and Crosses

To check the localization of Zipper in the cytoplasm of the terminal cells, *btl > gal4*, *UAS > cytoplasmic rfp* was obtained from Ghabrial Lab, while the Zip:GFP protein trap was obtained from the Vienna Stock collection, #115-082 [24]. The males possessing the *cytoplasmic rfp* were crossed with virgin females having *zipper gfp* driven by its endogenous promoter [25]. In order to create genetic mutations in the crosses to see the necessity of Zipper in branching morphogenesis, *btl > gal4*, *UAS > cytoplasmic gfp* was obtained from the Ghabrial Lab, while *UAS > zipper RNAi* was obtained from the Bloomington Stock Center, BL #65947 [24]. The virgin females had the gene for the *cytoplasmic gfp*, while the males had the gene for *zipper* RNAi [25].

### 2.2. Heat Kill

Heat kill was performed prior to confocal imaging in order to check branching and lumenogenesis patterns in the terminal cells of *D. melanogaster*’s tracheal system. Larvae were put in a drop of 60% glycerol on a glass slide. Then, the glass slide was placed on a 70 °C heat block for 5–10 s until larvae showed an instantaneous moment of vibration and was visibly dead. Then, the larvae were imaged with their dorsal side up [17].

### 2.3. Immunohistochemistry (Dissection/Fixation and Immunofluorescence/Mounting)

To check the localization of Zipper in the tracheal system, proper immunohistochemistry had to be performed. In a Sylguard pad full of ice-cold 1× PBS, larvae were pinned and cut with fine scissors on the ventral side. The body wall tissues were then spread out into an hexagonal shape with a pin on each of the six endpoints, and the internal organs were removed with fine forceps. The fillets were then fixed in 5 mL of 4% paraformaldehyde (PFA) for twenty minutes, incubated with primary antibodies overnight at 4 °C, and washed three times 15 min each at room temperature. Then, the fillets were incubated in secondary antibodies for one hour and washed three times 15 min each at room temperature. Samples were mounted in Aquapolymount and imaged on a Nikon C2 Confocal Microscope using NLS Elements Software [24,25]. For this particular experiment, the primary antibodies used were rabbit anti-RFP (1:1000 dilution, Rockland Immunochemicals, Inc. 600-401-379S) and mouse anti-GFP (1:1000 dilution, DSHB DSHB-GFP-12A6), while the secondary antibodies used were Alexa Fluor 568 donkey anti-rabbit IgG (1:1000 dilution, Thermoscientific A-10042) and Alexa Fluor 488 goat anti-mouse IgG (1:1000 dilution, Thermoscientific A-11001) [25]. These antibodies were used in order to amplify the signals of RFP and GFP. Although these signals are easily detected using confocal microscopy in native forms, they are heavily attenuated when endogenously expressed via genes inserted in model organisms [26]. Therefore, the antibodies were used to amplify the signals of the fluorescent proteins.

### 2.4. Qualitative and Quantitative Analysis

Branching and lumen analysis was performed on the dorsal branch terminal cells in the second tracheal metamere from the posterior of the first-generation third-instar heat-killed larvae. Samples were imaged on a Nikon C2 Confocal Microscope using NLS Elements Software [24]. Each branch in Z-stack images was traced using the Simple Neurite Tracer plugin from Fiji/ImageJ software. This led to a 2-dimensional image also to be used to check the branching pattern for each terminal cell. Sholl analysis was performed, and branching intersections were measured every 10 microns from the nucleus [25]. An original angle analysis was also performed, measuring the numerical value of the angle encompassing the branches for a terminal cell. The first line of the angle was fixed as the dividing line between the two terminal cells, while the second line of the angle encompassed the furthest visible branch from that terminal cell. For both Sholl and angle analyses, an F-test was performed to check for equal/unequal variance between the control and experimental samples. Following that, an equal/unequal variance independent 2-tailed T-test was performed to check for statistical significance in the data [27]. The T-test was performed at individual distances and as a whole data set for the Sholl analysis, and it was performed as a whole data set for the angle analysis.

### 2.5. Image Processing

All figures were prepared using the FigureJ plugin in Fiji using a published protocol [28]. When feasible, PowerPoint and R techniques were also used for figure preparations.

## 3. Results

### 3.1. Zipper Is Localized in the Cytoplasm of the D. melanogaster’s Terminal Cells

The first important test was checking the localization of Zipper. If Zipper is actually important for the branching in the terminal cells of the tracheal system, it is logical to hypothesize that it should be localized in or near the cells to have any effect in this process. Males with *btl > gal4*, *UAS > cytoplasmic rfp* were crossed with virgin females having *zipper gfp* driven by its endogenous promoter. This specific cross ensured that all F1-generation fruit flies had genes corresponding to both *cytoplasmic rfp* and *zipper gfp*. Then, the appropriate dissection/fixation and immunofluorescence/mounting protocol was performed. As shown in Figure 1A–C, there was a near-perfect merging of the cytoplasmic red with Zipper green, indicating the localization of Zipper in the cytoplasm of the terminal cell.

### 3.2. Zipper Is Necessary for Branching Morphogenesis in D. melanogaster’s Terminal Cells

In order to further test the importance of Zipper in branching morphogenesis of the terminal cells, the branches were visualized and compared between the wild-type and the RNAi mutants after heat-kill. The wild-type controls (Figure 2A–C) were simply an expression of the third dorsal terminal cells with *btl > gal4*, *UAS > cytoplasmic gfp*, while the experimental samples (Figure 2A’–C’) were an expression of the third dorsal terminal cell for the cross between the virgin female’s *btl > gal4*, *UAS > cytoplasmic gfp* and the male’s *btl > gal4*, *UAS > zipper RNAi*. The *zipper* RNAi terminal cells visibly showed less branching than their wild-type comparisons (Figure 2A–C’). More specifically, although there was a similar amount of branching close to the nucleus of each terminal cell, the amount of branching significantly decreased as one extends further out from the nucleus for the mutant tracheal cells.

To justify that the experimental terminal cells were true knockdowns of Zipper, a validation experiment was then performed using an alternative stock of mutants. More specifically, a new stock of virgin female with *btl > gal4*, *UAS > cytoplasmic gfp* was obtained from the Ghabrial Lab, while a new stock of male with *btl > gal4*, *UAS > zipper RNAi* was obtained from the Bloomington Stock Center. The knockdowns were then imaged (Figure 3A,B) using F1-crosses of the engineered genotypes. Similar to the first knockdown stock, there was a visible decrease in the amount of branching, particularly further away from the nucleus.

A rescue experiment was then performed using the samples in Figure 3 to demonstrate the sufficiency of Zipper in branching for *D. melanogaster*. These samples with the addition of Zipper are demonstrated in Figure 4. As shown, the fruit flies with rescued genotypes demonstrated similar phenotypes with wild-type fruit flies.

In order to make a quantifiable representation of the results encompassing the wild-types, RNAi knockdowns from various stocks, and rescued fruit flies, Sholl analysis was performed, counting the number of branches at every 50 μm from the nucleus. Interestingly, there was no statistically significant difference in the number of branches at distances equal to or less than 50 μm from the nucleus when measured in 10 μm increments. Nevertheless, there existed significant differences in the number of branches further away from the nucleus, suggesting that the initial propagation and lengthening of branches is not greatly affected by Zipper; nevertheless, at distal distances, the quantitative results hint at an essential role of Zipper in branching of the *D. melanogaster*’s terminal cells (Figure 5). An F-test value of *p* = 0.0023 indicated an unequal variance between the samples. An unequal variance independent 2-tailed T-test comparing the group of control and mutants in their entireties accumulating all values from 0 µm to 350 µm in 50 µm intervals generated a *p*-value of 0.0078 (Figure 5), indicating a statistically significant difference in the number of branches between the controls and the RNAi knockdowns as a whole dataset. The usage of an unequal variance 2-tailed T-test accounted for individual organism variability for all samples used in this analysis.

In order to make another validation as to Zipper’s role in branching in terminal cells, an original angle analysis was performed. More specifically, for each terminal cell, an angle checking the geometric distribution of the branches was calculated. By definition, an angle is the space between two intersecting lines, measured in units of degrees. For the purposes of the experiment, the first line of the angle was fixed as the dividing line between the two terminal cells, while the second line of the angle encompassed the furthest visible branch for the particular terminal cell (Figure 6A,B). The logic of this quantitative experiment was that should branching be hindered further away from the nucleus, the angle constructed by the constant line and the line encompassing the furthest branch would also be smaller, meaning this angle would be smaller for the mutants (Figure 6A,B), which demonstrated less branching further away from the nucleus in the aforementioned Sholl analysis. As deciding the two lines for each terminal cell was ambiguous at times, the same experimenter performed the angle analysis for all terminal cells to maintain consistency in the experimental procedure.

Parallel to the Sholl analysis data, the angle analysis data also showed smaller angles for the mutants compared to the controls, demonstrating the lack of geometric spread of the branches for the knockdowns (Table 1). The average angle for the controls was 109.65° with a standard deviation of 23.87°. On the other hand, the average angle for the mutants was 40.16° with a standard deviation of 24.66°. A F-test value of *p* = 0.79 means that these two sets of values virtually had equal variance and, therefore, individual-to-individual variability can be statistically neglected. The following equal variance independent 2-tailed T-test had a *p*-value of 0.00081 (<0.05), indicating a statistically significant difference in the numerical angles between the controls and mutants (Table 1). This matched the Sholl analysis results, which demonstrated less branching intersections for the mutant, especially as the distance from the nucleus of the terminal cell increased.

### 3.3. Zipper Is Not Necessary for Lumenogenesis in D. melanogaster’s Terminal Cells

Having shown that Zipper plays an important role in branching morphogenesis in the terminal cells of *D. melanogaster*, tests were performed to check whether Zipper also plays an important role in lumen formation. In this experiment, the same heat-kill and confocal imaging protocols were used where the lumen was visualized with a red stain, converted from a blue stain for clearer visualization. In this particular experiment, the lumen morphology was not visibly shown to be different between the controls (Figure 7A–C) and the experimental mutants (Figure 7A’–C’). What this indicated was that even with the absence of Zipper, proper lumenogenesis is possible, indicating that Zipper is not an essential component in lumen formation of the tracheal system. Considering the primary literature, which demonstrated no direct connection between Zipper and lumen formation [22], and noticing no significant visual difference in the lumens, a statement that Zipper does not play a significant role in seamless tube formation was made.

## 4. Discussion

First and foremost, the localization of Zipper in the cytoplasm of the terminal cell was shown, demonstrating that Zipper may play a role in the branching of the tracheal cells. Should Zipper not be shown to be localized in the cell, this may suggest that this particular protein does not play a direct role in branching morphogenesis. Nevertheless, seeing the localization in all tested samples indicated that the protein may play a role in branching within the model organism.

Further data elucidated that Zipper plays an essential role in the branching morphogenesis of the terminal cells in the tracheal system of *D. melanogaster*. More specifically, there was significantly less branching in the *zipper* RNAi samples compared to the wild-type, as demonstrated by both Sholl analysis and angle analysis. This result was found using *zipper* RNAi samples from two independent stocks. Furthermore, a rescue experiment using RNAi knockdown samples demonstrated phenotypes similar to those of wild-type fruit flies, thereby demonstrating the sufficiency of Zipper in branching morphogenesis. Nevertheless, Zipper was not shown to have a visible effect on the lumen formation within seamless tubes.

With such data in hand, the most rational role Zipper can play in branching morphogenesis is the regulation of filopodia formation. Bnl–Btl signaling leads to the extension of filopodia and lamellipodia, and branching follows in this direction of the FGF signaling [15]. The actin filaments need a myosin II’s actin-binding heavy chain, as this protein has contractile properties allowing cell adhesion and migration. What this ultimately suggests is that instigated by the Bnl–Btl signaling pathway, filopodia is extended via actin–Zipper interaction, which leads to cell elongation and respective branching. Therefore, in *zipper* RNAi mutants, the functioning of filopodia at branch tips is disrupted, hindering cell elongation and respective branching in the respective locations.

Interestingly, although there was less branching in the mutants, Sholl analysis indicated that there was no statistically significant difference in the number of branching intersections at distances equal to or less than 50 μm between the controls and knockdowns. What the data imply is that the major branches, hence those closer to the nucleus of the cell, are less affected by the presence and/or the absence of Zipper. This suggests that these proximal branches are already robust and fixed, meaning a lack of Zipper does not create detrimental effects. On the other hand, further away from the nucleus, cell growth is more dependent on filopodia. Hence, with a mutant *zipper*, there is no proper actin–Zipper interaction, therefore preventing cell migration and elongation, leading to a lack of respective branching in those regions. Thus, the sensitivity to filopodia and actin–Zipper interactions increases further away from the center of the cell and, hence, the nucleus.

For further investigation, one may ectopically inject incremental doses of Zipper in *zipper* null mutants, testing the dependency of filopodia at various distances from the nucleus of the cell. One may surmise that with more dependency on filopodia further away from the nucleus, one will require the highest dose of Zipper in these regions for there to be any sensible actin–Zipper interaction for cell elongation and branching. Nevertheless, it still remains uncertain whether filopodia formation is actually a key component in Zipper-dependent branching morphogenesis in the terminal cells of *D. melanogaster*.

Another experiment possible is biochemically testing in vitro what happens when a terminal cell is added with Bnl, Btl, actin, Zipper, and GFP tagging the cell’s cytoplasm. If further branching in the tracheal system is seen with the addition of only these components, this once again demonstrates the sufficiency of Zipper in promoting branching.

On the other hand, lumenogenesis appears to be unaffected by the lack of Zipper in RNAi mutants. Should *zipper* play a significant role in lumen formation, there must have been significant phenotypic differences in lumen formation between the controls and the mutants. Nevertheless, such differences were not noticeable, indicating that Zipper does not play an essential role in this particular process.

Hence, while Zipper appears to play a role in branching as a regulator of actin and apical polarity, there was no transparent evidence to support its role in lumen formation. However, it is still possible that Zipper plays a role in seamless tube formation, yet the dominating morphological defects in branching simply did not allow differences in lumen formation to be elucidated.

Moreover, the insignificance of Zipper in seamless tube formation does not justify that other myosin II’s actin-binding heavy chain do not play a role in the formation of seamless tubes. That said, it is critical to search for other genes responsible for lumen formation, possibly searching for other members in the myosin II’s actin-binding heavy chain group or in other domains such as the Rho GTPase family, including Cdc42, Rac1, and RhoA [29,30,31]. In fact, studying Rho proteins such as Cdc42 may provide another set of explanations as to how branching morphogenesis and lumenogenesis occur in the terminal cells of the *D. melanogaster*’s tracheal system.

More specifically, as a member of the PAR polarity complex that establishes apical/basal polarity in epithelial cells, Cdc42 is asymmetrically distributed and forms the axis for polarized growth, hence playing a critical role in establishing polarity [29]. Therefore, it is possible that Cdc42 plays a role in the formation and extension of filopodia, which is required for interaction with a myosin II’s actin-binding heavy chain and, hence, cell elongation; such a mechanism may pave a critical way for branching morphogenesis and/or lumen formation [32,33].

## 5. Conclusions

This paper was not able to compare functional phenotypes between wild-type and RNAi knockdown fruit flies, as these fruit flies were heat-killed and, thus, dead. However, morphological differences depicted by confocal microscopy provide hints as to how *D. melanogaster* lacking Zipper may behave compared to wild-type. Knowing that Zipper is necessary for branching morphogenesis of terminal cells in the tracheal system and utilizing the literature that branching morphogenesis is necessary for the transport of gases and metabolites [3], one may speculate that *zipper* mutants would lack transport of essential gases such as oxygen. This would debilitate the fruit fly’s respiratory track, naturally leading to its shorter life span.

As demonstrated by the results, there was no phenotypic difference in lumen formation patterns between wild-type and RNAi knockdowns. However, knowing that lumen forms via epithelial and endothelial tubes within the branched structures of the terminal cells [34,35], the fruit fly’s lumen phenotype can be considered to be masked by the branching phenotype. In other words, having an intact lumen is not helpful unless there is proper branching overarching the lumen, as the lumen forms after branching [12,13,14]. Therefore, should one try to predict the functionality of *D. melanogaster*’s tracheal system, it would be more effective to compare the functionality of branching of the terminal cells rather than comparing the functionality of lumen formation.

In short, this paper sought to check to role of Zipper in branching morphogenesis and lumenogenesis in the terminal cells of the *D. melanogaster*’s tracheal system. While no differences were found for lumen formation, qualitative and quantitative differences were found for branching between wild-types and RNAi knockdowns. This elucidated the fact that Zipper is necessary for branching morphogenesis, particularly in early developmental stages. A rescue experiment demonstrating how the addition of Zipper can revert the phenotype for RNAi knockdown mutants was helpful in suggesting that Zipper is sufficient for branching in the tracheal system of the fruit fly. Nevertheless, more research has to be carried out on Zipper and other myosin II’s actin-binding heavy chains to study the precise mechanism as to how development occurs within the terminal cells of the tracheal system for the *D. melanogaster*. Therefore, although this paper demonstrated Zipper’s role in the development of the terminal cells in the tracheal system, it is important to study how the protein is associated with other proteins in this regard.

## Figures and Tables

**Figure 1:** Localization of Zipper in cytoplasm. (**A**) is a merged photo of Zipper in the cytoplasm of the terminal cell in *Drosophila melanogaster*. (**B**) is a photo of the same terminal cell in *D. melanogaster* with only the cytoplasmic RFP signal. (**C**) demonstrates the same terminal cell with only the Zipper GFP signal.

**Figure 2:** Branching morphogenesis of controls and mutants. (**A**–**C**) represent the terminal cells of heat-killed third instar larvae for the controls, while (**A’**–**C’**) represent the experimental terminal cells of heat-killed larvae.

**Figure 3:** Branching morphogenesis of mutants from alternative stock. (**A**,**B**) represent the experimental terminal cells of heat-killed larvae using an alternative stock of fruit flies.

**Figure 4:** Branching morphogenesis of Zipper-rescued mutants from Figure 3. (**A**,**B**) represent the Zipper-rescued experimental terminal cells of heat-killed larvae using an alternative stock of fruit flies.

**Figure 5:** Sholl analysis for branching morphogenesis of controls and mutants. Sholl analysis demonstrated defective branching of RNAi mutants compared to wild-type with *n* = 40 for controls and *n* = 40 for mutants. The sample size represents the number of fruit flies that were used in the study. As only one terminal cell was observed for each fruit fly, the sample size also indicates the number of cells. Each fruit fly had a different and independent number of branches. Each of the branch measurements has been accounted for and included in the comparison between wild-types and RNAi mutants. Thus, this figure compares the controls and the mutants in their entireties at each distance from 0 µm to 350 µm in 50 µm intervals. The error bars show ± Standard Error of the Mean (SEM). Single asterisks (*) indicate *p* < 0.05, double asterisks (**) indicate *p* < 0.01, and no asterisk indicates no statistically significant difference in the pair of results when performing an equal/unequal variance independent two-tailed T-test. Whether to use an equal or unequal variance T-test was decided using a F-test, where *p* < 0.05 indicated unequal variance and *p* > 0.05 indicated equal variance. This process of checking for variance made sure to account for individual-to-individual organism variability for each incremental measurement.

**Figure 6:** Examples of angle° analysis for branching morphogenesis. The angle is indicated by the blue arc that is drawn between the first yellow line, which is a constant line intersecting the two terminal cells, and the second yellow line encompassing the furthest visible branch for the terminal cell of interest. (**A**) represents such an angle from a control, (**B**) represents such an angle from a RNAi knockdown.

**Figure 7:** Lumenogenesis of controls and mutants. (**A**–**C**) represent the lumens in the control cells. (**A’**–**C’**) represent lumens of the RNAi knockdown cells. The triangular structures represent denticles in the terminal cells irrelevant to the discussion of lumen formation.

**Table 1:** Angle° data for branching morphogenesis of controls and mutants.

	Cell 1	Cell 2	Cell 3	Cell 4	Cell 5	Cell 6
Control	78.68	124.64	93.40	102.59	146.30	112.30
Mutant	0.00	83.22	43.32	39.12	28.80	46.52

The first row indicates the angles for the controls with *n* = 6. The second row indicates the angles for mutants with *n* = 6. Similar to the Sholl analysis, the sample size for this angle analysis represents the number of organisms used in the study. As one terminal cell was analyzed for each organism, the sample size also represents the number of cells analyzed. Thus, the results of this table compares the controls and mutants in their entireties, concentrating on the angle for each sample based on the definition provided.

## Data Availability

Not applicable.
